# Application of AI Information Technology in the Political and Ideological Online Classroom System in the Background of Big Data

This article has been retracted.

**DOI:** 10.1155/2022/6590557

**Published:** 2022-07-08

**Authors:** Hao Wang, Jin Zhang

**Affiliations:** ^1^Department of Humanities and Foundation Courses, Shandong Polytechnic, Jinan, Shandong 250104, China; ^2^Yi'an Academy, Shandong Polytechnic, Jinan, Shandong 250104, China

## Abstract

Political and ideological online teaching is a new thing integrating political and ideological theory teaching and artificial intelligence information technology. In order to effectively improve the quality of political and ideological online teaching, this paper aims to make an in-depth study on the application of artificial intelligence technology in the political and ideological online classroom system under the background of big data. This paper first expounds the overall architecture of the political and ideological online system from the system hardware architecture and software architecture and then discusses in detail the functional design of the online system and the structure of the database. This paper proposes a data mining algorithm based on scale affine transformation and curriculum data information space reconstruction, constructs the data structure model of the political and ideological online classroom system, uses scale affine transformation to fuse the curriculum data, carries out spatial reconstruction of the fused curriculum data, extracts the high-order features of the curriculum data in the political and ideological online classroom system in the reconstructed space, and completes the data mining of political and ideological courses. Experiments show that the political and ideological online classroom system under the proposed method is better than the political and ideological online classroom system under the traditional method in terms of user satisfaction and teacher operation proficiency and can effectively improve the quality of political and ideological online teaching.

## 1. Introduction

Artificial intelligence (AI) is assumed as an interesting idea and a successful plan for the future lifestyle as it highly likely that most of the activities in those days will be carried out through the effective utilization of smart and intelligent robots. These robots may be equipped with sensors and actuator, where the former is used to interact directly with the phenomenon for which it is deployed to collect reading or data simultaneously. These sensors or devices are programmed such that it has the capabilities of automatically interacting and collecting data values after a defined time frame. Once the information is collected then it is processed inside the device by the concerned processing device to remove (if any) the noisy data value and then forward to the respective destination. For every activity, these intelligent robots are programmed such that when an abnormal condition, i.e., either the data value collect exceeds a particular threshold value or a slight decrease is measured, is encountered then actuator modules, which is embedded in an every device along with the sensors, takes the appropriate action which seems to be fit for that particular scenarios. As intelligence of these devices has a direct corelation with the smartness or intelligence of human beings, especially those who are going to program it, therefore, it is very important that these devices would mimic humans in performing various tasks, especially in the absence of human beings. These techniques are becoming more sophisticated and intelligent in terms of the decision when the concept of big data has been introduced and utilized in various domains.

In the context of big data, the independent learning of online courses and the coexistence of classroom special teaching and practical teaching inside and outside the class, the Trinity hybrid teaching mode has become the norm, and the effect of political and ideological teaching has been significantly improved. However, due to the weakening and marginalization of the discourse power of ideology, there are still difficulties in enhancing the construction and use of the political and ideological online curriculum system. For this reason, this paper makes considerable analysis and summary of the design ideas and the gap between the ideal and reality of the political and ideological online course system, and it puts forward perfect countermeasures. It is expected to effectively improve the quality of the political and ideological online classroom system, so that young students can share the high-quality resources of political and ideological education in the process of growth, achieve their all-round development in a diversified path, and highlight the significance of students' learning by using network resources.

According to the relevant national documents, combined with the ideological, political and theoretical characteristics, and talent training objectives, the online classroom teaching of political and ideological education needs to follow the curriculum design concept with students as the core, focus on the characteristics of political and ideological education on the basis of the unity of theoretical teaching and practical teaching, and adopt diversified online teaching methods and means to promote students from passive learning to active learning, improve the pertinence and timeliness of political and ideological online teaching, and enhance the absorption and appeal of the political and ideological online classroom, so as to improve students' learning enthusiasm and efficiency.

The innovations of this paper are as follows: (1) firstly, this paper expounds the system hardware architecture and software architecture, discusses in detail the functional design of the online system and the structure of the database, and puts forward a data mining algorithm based on scale affine transformation and curriculum data information space reconstruction to mine the political and ideological curriculum data. (2) Experiments show that the performance of the political and ideological online classroom system under the proposed method is better than that under other methods, and can effectively improve the quality of political and ideological online teaching.

The rest of the manuscript is as we have arranged it accordingly using a brief definition of various sections and subsections.

The most related or linked works to the problem at hand are reported with emphasis on whether these approaches are effective, i.e., in which scenarios, and have problems if these are applied to another domain for which it is assumed as one of the possible solution. The political and ideological online classroom system and its applicability in real world scenarios is reported along with sufficient detail information in section three of the manuscript. Research (preferably existing and related) on the political and online ideological classroom system based on artificial intelligence and information technology is reported in section four of the manuscript which is followed by analysis of the results, which were observed during the experimental setup, along with the textual explanation. Finally, a summary of the existing work along with a brief problem statement is presented in the last section of the paper.

## 2. Related Work

In recent years, China has paid more and more attention to network teaching, gradually attached importance to the research of the information-based political and ideological online classroom system, and achieved some results at the same time. Liu [1] with the gradual advancement of the new curriculum reform, many new teaching modes have been widely used. Among them, the mixed education mode has been comprehensively promoted in the current political and ideological teaching and achieved good results, as well as in political and ideological classroom teaching. However, there are many problems with the implementation of the mixed teaching mode in the political and ideological classroom. Therefore, we must pay great attention to it. On the basis of implementing the teaching mode of the political and ideological online classroom, we should effectively implement the mixed teaching mode, conduct in-depth research on the problems existing in the teaching process of the political and ideological online classroom system, and explore the construction way of the new political and ideological online classroom system, but this method does not improve the learning effect [1]. Aiming at the new concept of innovative teaching in the context of political and ideological education, Zhu et al. [2] have gradually become a new teaching norm. Therefore, this paper discusses the application value of the political and ideological online classroom system. Taking a university as an example, this paper studies the online teaching mode of political and ideological education, finds that the implementation of unit teaching is roughly divided into three stages, puts forward the design idea of the political and ideological classroom based on stages, and practices it. Through the implementation effect of political and ideological online courses, we can see that the overall implementation effect is relatively good, so as to realize the integration of knowledge transfer and value guidance, focus on the analysis of unreasonable problems, and putting forward improvement measures, but this method does not improve the quality of political and ideological teaching [2]. In the political and ideological online classroom, Yin and Zhang [3] separates the rights and obligations of instructors and students. The political and ideological online classroom's teaching approach is separated into two classes. The selection of a political and ideological online classroom teaching platform should be limited and improved, the educational goal should be gradual, the teaching process should be clear and smooth, and the evaluation of political and ideological classroom teaching should focus on effectiveness. Students must ensure active participation in political and ideological classroom discussions in order to improve political and ideological teachers' teaching ideas and operating skills, and to encourage students to realize generative dynamic independent construction in the learning process. The construction of Qiu [4] the political and ideological online classroom system aims to combine online teaching with classroom special teaching and practical teaching, creating a more distinctive mixed education mode of the political and ideological classroom, giving full play to the role of political and ideological teachers and students, and realizing the mutual penetration between political and ideological online classroom learning, classroom special teaching and practical teaching content inside and outside class, so as to realize the reform of curriculum assessment and evaluation. However, in the actual construction process, there are still some gaps with relevant requirements. Schools, teachers, and students cannot reach a consensus, resulting in poor learning efficiency of students and failure to play an important role of the political and ideological online classroom system [4].

## 3. Political and Ideological Online Classroom System

### 3.1. Framework Design of the Political and Ideological Online Classroom System

1. The topology of the political and ideological online classroom system server is shown in Figure 1. The overall system includes web server, mail server, directory server, and database server [5, 6].
2. The network architecture system in Figure 1 has a hardware structure that comprises an interface server, a database server, a web server, and a student side module, among other things. Figure 1 shows the database server at the heart of the political and ideological online classroom system. It can gather a variety of political and ideological theory data and interchange it with a remote server, allowing for the upload of political and ideological theory data as well as the download of instructions. Web server is the software logic of the political and ideological online classroom system. This server uses Iis7.0 and other management applications to conduct software operations. The web server is connected to the system from the network. The student side logs in to the online classroom system from the network and accesses the request to the web server. The service area performs specific services and then returns to the results. The student terminal has a unique function: it is a terminal for local operation. The student terminal talks with the server and transfers data across the network to the background processing center. The student terminal may also accept data supplied from a remote location, convert it to local format, and deliver it to the server [7, 8].
3. The system integration architecture of the political and ideological online classroom is mainly divided into UI layer, service layer, and persistence layer, which is shown in Figure 2. In Figure 2, the UI layer includes the user authentication portal and the service platform. The management platform mainly adopts user authorization management and a single sign on the system management platform. The service layer is based on the digital certificate identity authentication system and supports password and certificate login. The single sign-on service supports the B/S architecture, supports many student terminals, provides the single sign-on mode of reverse proxy, and supports cross-regional single sign-on. Student authorization service refers to that the administrator can use the open interface of the business system to obtain the function module and role data of the corresponding business system, and carry out permission allocation to users. The persistence layer is mainly used for configuration information storage, which is mostly used for later audit. The main functions of the political and ideological online classroom system focus on managing the information resources of organizations, users, and application systems, and providing identity authentication and authorization services for the political and ideological online classroom system [9, 10].

### 3.2. Function Design of the political and Ideological Online Classroom System

#### 3.2.1. Function Design of the Slide in Political and Ideological Course

The functional module of the political and ideological course slide is shown in Figure 3. The slide management of political and ideological course in Figure 3 can complete students' slide management of political and ideological course. The slide management of political and ideological course is mainly divided into the teacher course slide and the student course slide. We input the slides corresponding to each chapter of political and ideological course into the political and ideological online classroom system, including the time, title, content, and reporter of the course slides. Through the role module setting, in the role module, only political and ideological teachers can maintain the course slides, while students can only query the course slides. Students' course slides are the slides corresponding to the course learning input into the political and ideological online classroom system, including the time, title, content of the course slides, submitter, and introduction. Through the setting of the role module, in the role module, political and ideological teachers can maintain the course slides, while students can only manage the course slides [11, 12].

#### 3.2.2. Video Function Design of the Political and Ideological Online Classroom

The main function of political and ideological course video management is to configure and manage the video information of political and ideological course in teaching. The functions of political and ideological course video management include creating the political and ideological course video, deleting the political and ideological course video, and modifying the political and ideological course video. Through the role module setting, only political and ideological teachers in the role module can maintain course video information, and other users can only query the political and ideological course video.

#### 3.2.3. Design of Feedback Management Function of Political and Ideological Course

In the process of learning political and ideological education, students can send questions to the political and ideological education teacher after the class, and the teacher will reply after seeing the questions. This can not only improve the teaching quality, but also facilitate the communication efficiency. It is a very important function in the online classroom teaching system.

#### 3.2.4. In Political and Ideological Courses, the Functional Design of Test Question Management

The primary goal of political and ideological classroom test question management is to look at certain chapters of political and ideological education. The report of course test questions, the compilation of course test questions, and the alteration of course test questions are all functions of political and ideological course test question management. Only political and ideological teachers may maintain course video information using role module configuration, while students can only query the political and ideological course test questions [13, 14].

#### 3.2.5. Function Design of Online Discussion of Political and Ideological Course

Figure 4 shows the specific functional modules of online discussion management. In Figure 4, the online discussion function refers to the online discussion carried out by teachers in Political & ideological teaching. The functions of online discussion management include opening and closing the discussion area, answering questions and publishing discussions.

### 3.3. Structure Design of System Database Table

The political and ideological online classroom system in this paper has high requirements for database security, and the amount of data in the design is relatively large, which also has requirements for the size of the database. Therefore, a large database with a high level is adopted, and an SQL server is used as the platform of the system database. Tables 1 and 2 represent the student table and teacher table, respectively. The student attributes include student name, student password, e-mail address, and nickname picture. Teacher attributes include teacher name, teacher password, e-mail address, and nickname picture [15, 16].

## 4. Online Political and Ideological Classroom System Based on Artificial Intelligence and Information Technology

Combined with the above political and ideological online classroom system, the data mining algorithm based on scale affine transformation and data flow spatial reconstruction is used to study the political and ideological online classroom system.

In the political and ideological online classroom system, we perform adaptive learning on the attribute weight of the data storage model, and we build the particular data distribution vector field of the political and ideological course database in the multilayer vector regression feature space. Local outliers will produce a cross-course data set in the political and ideological online classroom system. We use formula (1) to construct the information model of local outliers in the data mining of specific political and ideological courses, which is expressed as

(1) $$\begin{array}{c} D_{w}\left(s\right)=\frac{\sum_{u,v\in S}V_{M_{i}}}{\left|S\right|\times \left(\left(\left|S\right|-1\right)/2\right)}. \end{array}$$

In formula (1), *w*_*u*,*v*_ represent the weights between network nodes *u* and *v* in the political and ideological online classroom system, and |*S*| represents the cross points of the course data characteristics in the undirected graph *S*.

Formula (2) is used to express the distribution probability of specific data in *k* political and ideological online classroom systems evenly distributed in the data edge subband as

(2) $$\begin{array}{c} p_{k}=\left[\begin{array}{c} N-1\\ k \end{array}\right]p_{2\;D}^{k}{\left(1-p_{20}\right)}^{N-1-K},\;k=0,1,2,\ldots ,N. \end{array}$$

According to the distribution probability of the specific data of the political and ideological online classroom system, the scale affine transformation is carried out on the course data with large distribution probability, and the political and ideological course information fusion model of data mining with a limited signal-to-noise ratio is constructed, which is expressed as

(3) $$\begin{array}{c} \psi_{a,b}\left(t\right)=\left[U\left(a,b\right)\psi \left(t\right)\right]\\ =\frac{1}{\sqrt{\left|a\right|}}\psi \left(\frac{t-b}{a}\right). \end{array}$$

In formula (3), *U*(*a*, *b*) represents the Fourier transform of the time domain part of the specific course data in the political and ideological online classroom system, and the factor $1/\sqrt{\left|a\right|}$ ensures the normalization of the Fourier transform energy. After the processing of the above process, the course data information fusion in the political and ideological online classroom system is realized [17, 18].

Assuming the optimal weight coefficient *β* and the penalty factor *C* of the curriculum data fusion in the political and ideological online classroom system, the mean square deviation function of gain adjustment of curriculum data is established by formula (4), which is expressed as

(4) $$\begin{array}{c} F_{\text{fitness}}=\frac{1}{m}\sum_{i=1}^{m}{\left(\beta -C\right)}^{2}. \end{array}$$

A multi distributed database model is used to manage course data in the political and ideological online classroom system. The distributed database contains a large number of course data. The gain adjusted mean square deviation function must be used to optimize the course data in the political and ideological online classroom system, so as to improve the accuracy and efficiency of course data mining, Decompose the attenuation characteristics of specific course data information through the spatial reconstruction method of the following formula:

(5) $$\begin{array}{c} x\left(t\right)=f\left(x\left(t-1\right),W^{11}x\left(t-1\right),W^{21}x\left(t-1\right)\right)\\ \varepsilon \left(t-1\right),W^{11}\eta \left(t-1\right),W^{21}\varepsilon \left(t-1\right). \end{array}$$

After the decomposition of attenuation characteristics is completed, the directional characteristics of the curriculum data in the political and ideological online classroom system are adopted, and the nonuniform sampling output of the response characteristics of the curriculum data in the political and ideological online classroom system is obtained by the following formula:

(6) $$\begin{array}{c} {\hat{f}}_{i}\left(t,\tau \right)=\frac{1}{2\pi \tau }\sum_{k=-q/2}^{q/2}b_{k}\phi x\left(t\right). \end{array}$$

In formula (6), *τ* represents the sampling delay raised in the data information space of a specific course, and *ϕ* represents the phase difference of data sampling interval. Obtain the characteristics of political and ideological course (time shift) through the following formula:

(7) $$\begin{array}{c} \left\{\begin{array}{c} y\left(t\right)=x\left(t-t_{0}\right)\Rightarrow W_{y}\left(r,v\right)=W_{x}\left(t-t_{0},v\right),\\ y\left(t\right)=x\left(t\right)e^{j2\pi v_{0}t}\Rightarrow W_{y}\left(t,v\right)=W_{x}\left(t,v-v_{0}\right). \end{array}\right. \end{array}$$

In formula (7), *x*(*t*) represents the decomposition result of the original course data, *t*_0_ represents the time point of the initial sampling of the data, *W*_*y*_(*t*, *v*) represents the observed vector, *v*_0_ represents the specific data density of course, and *v* represents the interference intensity of the data in the online classroom system. The matrix *X*(*i*) of the course data information fusion in the political and ideological online classroom system is divided into *p*(*i*) spatial matrix *X*_*ij*_. The matrix *X*_*ij*_ in the *j* subspace is reconstructed in high-dimensional space by formula (8), and the singular value decomposition is expressed as

(8) $$\begin{array}{c} \min_{\beta }\left\|Y\left(i\right)-X\left(i\right)\beta \right\|=\min_{\beta }\left\|U_{i1}^{\prime T}Y_{i1}-\sum_{i1}^{\prime }V_{i1}^{\prime T}\beta \right\|. \end{array}$$

After singular value decomposition, the higher-order features of curriculum data in the political and ideological online curriculum system are extracted from the curriculum data reconstruction space through formula (9) and expressed as

(9) $$\begin{array}{c} \min_{\beta }\left\|Y\left(i\right)-X\left(i\right)\beta \right\|=\min_{\beta }\left\|\left[\begin{array}{c} Y_{i1}\\ Y_{i2}\\ M\\ Y_{ip\left(i\right)} \end{array}\right]-U\left(i\right)\left[\begin{array}{c} \sum_{it}V_{it}^{T}\\ \sum_{i2}V_{i2}^{T}\\ M\\ \sum_{ip\left(i\right)}V_{ip\left(i\right)}^{T} \end{array}\right]\beta \right\|. \end{array}$$

Among them, the high-order features of course data in the political and ideological online classroom system can reflect the characteristics of course data to a certain extent. By positioning the high-order features, the course data mining in the political and ideological online classroom system can be realized [19, 20].

## 5. Analysis of Experimental Results

In order to effectively verify the performance of the political and ideological online classroom system based on artificial intelligence information technology under big data, experimental verification is carried out.  Table 3 shows the hardware configuration statistics of the political and ideological online classroom system. The function configuration of the political and ideological online classroom system, and the function provided by the web is IIS7.0. The software service of the database is SQL server2018 and the test terminal is IE8.0.

Table 2 represents the comparison of course data mining time between the political and ideological online classroom system based on artificial intelligence information technology and the traditional political and ideological online classroom system.

As can be seen from the data in Table 4, when compared to the course data mining time of traditional methods, the method proposed in this paper has a short data mining time, allowing it to quickly find the key contents of political and ideological online classroom teaching, thereby improving learning efficiency. This study chooses 50 professors and 50 students from a university for 300 hours of online instruction and compares the satisfaction and competency of the political and ideological online classroom system using the approach provided in this research to other methods.  Figure 5 shows the satisfaction comparison between the political and ideological online classroom system of the method proposed in the text and the political and ideological online classroom system of the traditional method.

By analyzing the data in Figure 5, we can see that the use satisfaction of the political and ideological online classroom system under the traditional method is low from the initial stage. With the increase of the number of times of system use, the use satisfaction does not fluctuate much, and it continues to be in a low state. The use satisfaction of the political and ideological online classroom system under the method proposed in this paper is higher from the perspective of the initial satisfaction of the system. With the gradual increase of the use times of the system, the satisfaction has been very stable, because the method proposed in this paper adopts the data mining algorithm of scale affine transformation and data flow space reconstruction, which can quickly mine the relevant course data needed in the classroom, improving the efficiency of teaching, and improving the satisfaction of the use of the system.  Figure 6 shows the proficiency comparison between the proposed method and the traditional method.

Through the analysis of Figure 6, it can be seen that teachers' proficiency in the operation of the political and ideological online classroom system under the traditional method is poor from the beginning. With the gradual increase of use times, the operation proficiency also increases, but it is not high on the whole, indicating that although the use times increase, the overall operation proficiency is poor. Teachers' operation proficiency of the political and ideological online classroom system of the method proposed in this paper is obviously improved with the gradual increase of the use times. This shows that the online system using the method proposed in this paper can effectively improve the efficiency of teaching, so as to enhance students' learning enthusiasm.  Figure 7 shows the comparison of the fault tolerance rate of the political and ideological online classroom system under the proposed method and the traditional method.

The analysis of Figure 7 shows that the fault tolerance rate of the political and ideological online course system under the proposed method is low, which shows that it has a little impact on the use effect of the political and ideological online classroom system, and the use of the system under the proposed method can effectively improve the teaching quality of teachers. The fault tolerance rate of the online political and ideological course system under the traditional method is relatively good, which will have a great impact on the use effect of the online political and ideological classroom system, resulting in the poor use effect of the online political and ideological classroom system under the traditional method, which reduces the efficiency and quality of teachers' teaching.

## 6. Conclusion

The application of the political and ideological online classroom system accumulates experience for the improvement of teaching quality of political and ideological education. Although the political and ideological online classroom system still has some deficiencies in the practice of online teaching, it can effectively promote the reform of political and ideological courses in colleges and universities and the application and development of mixed mode teaching. The political and ideological theory online teaching system is a relatively huge project. The teaching management department must work together with the student work department and the society to strengthen the interaction between teaching and learning and improve the political and ideological online classroom system, effectively grasp the dynamics of students' learning. As proved from the observation of the results in terms various metrics, the proposed scheme is an effective solution to resolve the problem at hand, especially with the available resources and infrastructures.

## Figures and Tables

**Figure 1:** Topological structure of the political and ideological online classroom system server.

**Figure 2:** System software architecture diagram.

**Figure 3:** Functional modules of the political and ideological course slide.

**Figure 4:** Specific functional modules of online discussion management.

**Figure 5:** Comparison of the satisfaction of using the political and ideological online classroom system in different methods.

**Figure 6:** Comparison of teachers' operating system proficiency under different methods.

**Figure 7:** Comparison of the fault tolerance rate of the political and ideological online course system under different methods.

**Table 1:** Student table.

Data entry name	Table item type	The value can be null	Primary key/foreign key
Since the primary key	Int	Do not empty	Since the primary key
The student name	Var-char (50)	Do not empty	
Student password	Var-char (50)	Do not empty	
E-mail address	Var-char (50)	Do not empty	
Nickname	Var-char (50)	Can be null	
The picture	Binary	Can be null	

**Table 2:** Teacher table.

Data entry name	Table item type	The default value can be null	Primary key/foreign key
Since the primary key	Int	Do not empty	Since the primary key
The teacher name	Var-char (50)	Do not empty	
The teacher password	Var-char (50)	Do not empty	
E-mail address	Var-char (50)	Do not empty	
Nickname	Var-char (50)	Can be null	
The picture	Binary	Can be null	

**Table 3:** Hardware Configuration of the Political and ideological Online Classroom System.

	CPU	Storage capacity (G)	The hard disk (G)	The operating system
The web server	Intel core i7-4712MQ	8	160	Windows 7
Database server	Intel core i7-4712MQ	8	320	Windows 7
The test terminal	Intel core i3	4	160	Windows 7

**Table 4:** Comparison of system data mining time under different methods.

Methods	Data mining time (ms)
In this paper, methods	15
The traditional method	26

## Data Availability

The datasets used during the present study are available from the corresponding author upon reasonable request.
